# Application Research of Artificial Intelligence Screening System for Diabetic Retinopathy

**DOI:** 10.1155/2022/2185547

**Published:** 2022-01-17

**Authors:** Yuwen Wang, Lina Wang, Heding Zhou, Yanhong Liao, Quanyong Yi

**Affiliations:** ^1^Ophthalmology Department, Ningbo Eye Hospital, Ningbo 315040, China; ^2^Department of Information, Ningbo Eye Hospital, Ningbo 315040, China

## Abstract

According to the latest data from the Bureau of Disease Control and Prevention of the National Health and Family Planning Commission, China currently has 199.6 million diabetic patients and has become the world's largest country with diabetes. The prevalence rate is as high as 14.3%, which is much higher than the world average of 5.8%. The primary-level ophthalmic screening service is one of the important tasks to improve primary-level medical services, and the corresponding ophthalmic imaging diagnosis technology is an important support for primary-level medical and health services. Therefore, it is very necessary for us to study the application of artificial intelligence image recognition technology for diabetic retinopathy under the medical consortium mode and to study the precise initial diagnosis, precise referral, and precise follow-up of diabetic retina under the medical conjoined mode, so as to better promote the transformation of the ophthalmology primary service model. Based on this background, in this article, we have proposed and carried out the following solution: (1) diabetes data collation. Based on medical artificial intelligence technology, this paper collected 2,265 electronic medical records from an eye hospital in Ningbo and selected 2,000 qualified medical records for data integration and preprocessing. The contents of electronic medical records mainly include age, gender, and examination records. (2) Establish diabetic retinopathy diagnosis model based on neural network algorithm. This article first uses the classic algorithm of BP neural network for modeling, chooses the Levenberg–Marquardt method as the training function, and selects 10 hidden layer units through comparison experiments. After that, ophthalmologists assessed 80 sets of test results and determined the right diagnosis rate. Finally, this article compares and analyzes the accuracy of the two routes in 80 tests.

## 1. Introduction

As people's living circumstances improve, the number of diabetics increases dramatically [1, 2]. It is not uncommon for diabetics to develop complications like diabetic retinopathy, a common retinal vascular disease, and a major cause of blindness in diabetic patients. Because there are often no clinical symptoms in the early stage of DR, and once there are symptoms, the condition is already serious and it is easy to miss the best treatment time [3]. Blindness caused by DR accounts for about 8%–12% of all blind patients, and the probability of blindness in China is about 25 times that of nondiabetic patients [4]. Early screening, early diagnosis, and early treatment are the keys to preserving vision in patients with DR. As of 2017, there are more than 30 million DR patients in China, 70% of whom have not received standardized treatment [5]. Compared with the huge number of patients, there is a serious shortage of ophthalmologists in China. According to the statistics of the National Health and Family Planning Commission, there are currently only 36,000 ophthalmologists in China, of which less than 10,000 doctors are engaged in fundus medical services and research. The ratio is less than 10%. Through regular screening of fundus lesions and early diagnosis, nearly 90% of visual impairment and blindness induced by diabetes can be completely avoided [6]. However, in recent years, the country has paid increasing attention to the prevention and treatment of diabetes and its complications. On April 11, 2017, the General Office of the National Health Commission issued a notice on the issuance of the technical plan for the graded diagnosis and treatment of diabetic retinopathy. It is required to achieve early detection and early intervention of DR to reduce the disease burden of the people. The development of the medical consortium model has resulted in a significant increase in the number of screening tasks for diabetic retina being gradually assigned to ophthalmologists in primary hospitals and general practitioners in community health service centers， with the number of tasks increasing year after year and the severity of the screening tasks becoming more severe. The traditional methods of screening for DR include direct ophthalmoscope, fundus color photography, fundus angiography, etc., while fundus color photography is a simple and efficient method for screening fundus diseases, which is generally considered to be the most suitable for screening and follow-up [7–9].

However, with the increase in the number of people with diabetes and the lack of ophthalmologists, the traditional concept of DR screening methods cannot effectively cope with the dual challenges of increasing DR prevalence and blindness. At the same time, it is a highly professional task to determine whether there is a GlycoNet in fundus photographs, and it is usually difficult for general practitioners, internal medicine physicians, and even endocrinologists to do the job. At the same time, the “Opinions on Deepening the Reform of the Medical and Health System” of the Health and Family Planning Commission also clarified the construction ideas of “using network information technology to promote the cooperation between urban hospitals and social health service agencies,” and established the integration of regional resources and the construction of regional health services. The “Opinions on Deepening the Reform of the Medical and Health System” also emphasizes the need to change the service model, to “strengthen the grassroots, build mechanisms, and encourage diversified medical services.” Promoting the process of “double sinking and two upgrading” is a problem that we urgently need to solve.

In this article, artificial intelligence screening system for diabetic retinopathy has been presented which has the following tasks:

- Verify the accuracy of artificial intelligence technology in diagnosing DR detection under the equipment and operating mode of this subject
- Analyze the operating efficiency, awareness, and satisfaction of the DR artificial intelligence screening system in Ningbo based on the medical consortium model, and evaluate its actual operating effects
- Through the operation of DR artificial intelligence screening mode, improve the diagnosis level of community doctors in ophthalmology, which will help promote the mutual cooperation of all levels of hospitals in the medical system, promote the vertical integration of urban and rural medical resources, and sink high-quality medical resources
- Through the analysis of a large sample of screening data, we can draw conclusions about the relationship between the prevalence of DR patients in Ningbo area and factors such as age, environment, gender, as well as the distribution of DR patients in Ningbo area, and the degree of disease classification, etc., to provide government departments with decision-making, and it provides new clinical and basic research directions for the occurrence and development of DR
- Actively promote the clinical application of high-tech in the medical field, and expand the application of interdisciplinary
- Use the application of artificial intelligence technology in DR detection to explore the establishment and improvement of the Ningbo DR screening model, improve screening efficiency, expand coverage, so that patients can get treatment in time, and effectively reduce the number of blindness caused by DR in Ningbo

The remaining paper is organized as follows. In the subsequent section, a detailed description and analysis of the existing state-of-the-art mechanism are presented which followed by the description of the proposed method. Then, a comprehensive analysis of the proposed method and its effectiveness in resolving the aforementioned issues is presented. Experimental results are thoroughly examined and explained with proper justification in the experimental results section. Finally, concluding remarks and future direction are given.

## 2. Related Work

Many diabetic retina screening responsibilities have been steadily assigned to ophthalmologists in primary hospitals and general practitioners in community health service centers with the growth of the medical consortium model, and these tasks will increase year on year and become more severe. Traditional DR screening methods include direct ophthalmoscope, fundus color photography, fundus angiography, etc., while fundus color photography is a simple and efficient screening method for fundus diseases, which is generally considered to be the most suitable for DR screening and follow-up. However, with the increase in the number of people with diabetes and the lack of ophthalmologists, the traditional concept of DR screening methods cannot effectively cope with the dual challenges of increasing DR prevalence and blindness. At the same time, it is a highly professional task to determine whether there is a GlycoNet in fundus photographs, and it is usually difficult for general practitioners, internal medicine physicians, and even endocrinologists to do the job. At the same time, the “Opinions on Deepening the Reform of the Medical and Health System” of the Health and Family Planning Commission also clarified the construction ideas of “using network information technology to promote the cooperation between urban hospitals and social health service agencies,” and established the integration of regional resources and the construction of regional health services. The “Opinions on Deepening the Reform of the Medical and Health System” also emphasizes the need to change the service model, to “strengthen the grassroots, build mechanisms, and encourage diversified medical services.” The primary-level ophthalmic screening service is one of the important tasks to improve primary-level medical services, and the corresponding ophthalmic imaging diagnosis technology is an important support for primary-level medical and health services [10].

After years of working with Google TensorFlow and Inception V3 models for training, the Google DeepMind team presented an AI screening study for diabetic retinopathy in 2016, and eventually, the accuracy of AI diagnosis was better than that of ophthalmologists [11]. Congenital cataract is a rare eye disease. The team of Haotian Lin from Sun Yat-sen University's Ophthalmology Center and Liu Xiyang from Xidian University used only a small number of samples to preprocess the image using methods such as Hough transform to extract the region of interest, then transfer learning method is based on the Caffe and AlexNet model for training, the final diagnosis accuracy reaches the level of experts, and the cloud screening and diagnosis platform CCCruiser are established, which improves the coverage of high-quality medical resources [12]. In April of this year, the system went live. There has been a steady stream of AI results for the automatic detection of eye disorders since then [13]. Global fundus disease screening systems were released in 2017 that are multiethnic and multicenter. Since then, a closed diagnostic circuit has developed for fundus illnesses, and it has met the required standards for clinical use [14]. In 2018, Zhang Kang's team used Google TensorFlow and Inception V3 models to select 108,312 two-dimensional tomographic images from 4686 patients' ocular optical coherence tomography (OCT) data for model training. The results showed that it can effectively diagnose macular degeneration and diabetic retina disease has also reached the level of experts [15]. Image processing and analysis methods have undergone radical changes thanks to advances in deep learning technology, which has enabled researchers to identify phenomena they had never seen before [16]. For the first time in 2018, the DeepMind team at Google utilized fundus pictures and deep learning to accurately forecast the risk of heart disease [17]. IDx's AI diabetic retinopathy clinical diagnosis system was examined by the US Food and Drug Administration at the same time [18], which brings it one step closer to being approved for formal clinical use. The essence of artificial intelligence image recognition technology for diabetic retina is a computer deep learning algorithm. The accuracy of diagnosing DR under laboratory conditions has exceeded 99%, far exceeding the average level of human ophthalmologists, and even exceeding the diagnosis level of ophthalmologists. Using artificial intelligence technology, after pretraining, the level of DR diagnosis basically reaches the level of fundus doctors, and the work efficiency is much higher than that of human doctors [19]. Many domestic scientific research units have been engaged in related research work [20–25], and some attempts have been made in the field of DR screening, but there are few reports on the application of large sample sizes in real scenarios and in the medical consortium model. At the same time, although there have been precedents for sugar network screening using artificial intelligence technology across the country, such as Beijing Tongren Hospital, Zhejiang Eye Hospital, Jing'an District Northern Medical Community, 51 community health service centers in the main urban area of Hangzhou, etc., Ningbo has not yet launched a similar project. At the same time, there is no report on the research of fundus image quality evaluation, big data analysis, grassroots image reading assessment, operation efficiency evaluation, Ningbo market prospects, and evaluation of the output value of related follow-up services driven by screening.

## 3. Proposed Methodology

### 3.1. Principle of Neural Network

The mathematical model of artificial neural network (ANN) for information processing is similar to the connection structure of the neural synapses of the human brain. A large number of nodes (“neurons” or “units”) are connected to each other to form the basic network of the neural network model. Neural networks can only be used after training. The training of the network is the process of network self-learning. The training changes the connection weights of the network nodes, so that it has a classification function, and can be used for object recognition in the end. The advantages of neural networks are as follows: (1) neural networks can approximate arbitrary functions with arbitrary precision; (2) neural networks can handle various complex data relationships due to their own nonlinear model properties; (3) neural networks are compared to other classification algorithms, and its powerful learning ability enables it to better adapt to changes in the data space; (4) neural networks are constructed by pulling inspiration from the human brain in order to mimic some of the brain's capabilities and realize their full Internet meaning of the word “smart.” Scientists inspired ANN research when trying to simulate the biological nervous system. Neurons, the brain's primary building block, are linked by filaments known as axons, which run throughout the brain. When neurons are stimulated, nerve impulses are transmitted from one neuron to another through axons. Dendrites are extensions of neuron cells. A certain neuron connects to the axons of other neurons through the dendrites. The connection points between dendrites and axons are called nerve bonds. Neuroscientists have discovered through research that under the repeated stimulation of the same pulse, the strength of the connection of the nerve bonds between neurons will change, and the human brain will learn through this process. According to the different topological structures, the neural network can be divided into a forward network and a feedback network.

#### 3.1.1. Forward Network

This is a network that only contains an input layer and an output layer, as shown in Figure 1. A node is a neuron, and there is no connection between nodes in the same layer. Neurons' transfer function is usually a sigmoid-type function. Sometimes, a linear function is selected as the neuron transfer function of the input layer or output layer. This network is usually used for linear classification.

#### 3.1.2. Feedback Network

The input data determine the starting state of the feedback network of a system using a neural network feedback mechanism. After a series of state transitions, if the system can gradually converge to a stable state, then this stable state is the calculated output of the feedback neural network result. This design is to make the network finally reach a stable state through feedback calculation under the initial input, and its output point is the balance point that the user needs.

### 3.2. BP Neural Network

The back propagation (BP) neural network is a multilayer feedforward neural network that works by forwarding the input signal and solving the weight adjustment problem by propagating the error signal backward while it is in use. BP neural network input vector propagates forward from input layer neurons to hidden layer neurons, where it is processed and transformed before being sent to the output layer via a synergy of weights, thresholds, and transfer functions. The number of hidden layers can be dynamically adjusted to meet the actual data processing needs, and the output layer will then output. BP networks transfer output value differences backward from the output layer to the hidden layer and to the input layer, which is known as back propagation. Each layer's weights and thresholds will be adjusted as the process progresses. We refer to the training and learning process of neural networks as the gradual change of network parameters via forward and backward propagation. A network training process will come to an end whenever the set error range is reached during the learning phase. Input and output, transfer function, error computation, and self-learning are all parts of the BP neural network structure. The following are their formulations for spatial state:

(1) Hidden layer node output:
  (1) $$\begin{array}{c} O_{j}=f\left(\sum \omega_{ij}x_{i}-q_{j}\right), \end{array}$$
where *q*_*j*_ is the threshold of the hidden layer.
(2) Output layer node output:
  (2) $$\begin{array}{c} O_{k}=f\left(\sum \omega_{jk}O_{j}-b_{k}\right), \end{array}$$
where *b*_*k*_ is the threshold of the output layer.
(3) Also known as stimulus function, a continuous sigmoid with value range (-1,1) or (0,1) serves as the transfer function, which reflects the degree of intensity and mode of action between the two node layers:
  (3) $$\begin{array}{c} \left\{\begin{array}{c} \log\text{ sig}\left(n\right)=\frac{1}{\left(1+\exp\left(-n\right)\right)},\\ \tan\text{ sig}\left(n\right)=\frac{2}{1+\exp\left(-2n\right)}-1. \end{array}\right. \end{array}$$
(4) The network uses formula (4) to calculate the error between the output and the actual output of the data:
  (4) $$\begin{array}{c} E=\frac{1}{2}\sum {\left(T_{k}-O_{k}\right)}^{2}, \end{array}$$
where *T*_*k*_ represents the actual output value of the data and *O*_*k*_ represents the calculated output value of the network.
(5) A crucial function in the BP neural network is being carried out by the self-learning component, which is constantly modifying the initial weights and error feedback between the higher and lower nodes. The model is as follows:
  (5) $$\begin{array}{c} \omega_{ij}\left(n+1\right)=h\times \phi_{i}\times O_{k}+\alpha \times \omega_{ij}\left(n\right), \end{array}$$
where *ω*_*ij*_ is the connection weight between two adjacent layers; *h* is the learning factor; *ϕ*_*i*_ is the calculation error of the output node; *O*_*k*_ is the calculation output of the output node; and *α* is the momentum factor. The mapping capability of the BP neural network to transfer input values to output may accomplish any complex nonlinear mapping function after mathematical proof.

### 3.3. Preliminary Assessment

Group comparison to verify the accuracy of artificial intelligence diagnosis collected 2265 patient information from Ningbo Eye Hospital and screened out a total of 2,000 qualified research subjects. Compose high-quality fundus photos into a test data set, submit them to artificial intelligence technology and fundus disease specialists for diagnosis, and compare the accuracy of the two. Diagnose and classify each image according to the international DR staging standard: (1) no diabetic retinopathy; (2) mild nonvalue-added diabetic retinopathy; (3) moderate nonvalue-added diabetic retinopathy; (4) severe nonvalue-added diabetic retinopathy; and (5) proliferative diabetic retinopathy. Based on the five-category model, the same experienced Ningbo Eye Hospital ophthalmologist will evaluate the fundus photos of the test data set separately, divide the fundus photos into 5 levels according to the severity of DR, and then use the trained artificial intelligence model to test the fundus photos of the data set which are divided into 5 levels to evaluate the accuracy of the algorithm model. If the accuracy of artificial intelligence diagnosis is higher than 95%, it is considered that the actual application conditions are met. Otherwise, large sample mark training is used until the diagnosis accuracy of the artificial intelligence model meets the requirements. The technical route of the research is shown in Figure 2:

### 3.4. Comparing the Evaluation Indicators of the Two Paths

Based on the preliminary establishment of the regional specialist medical consortium screening system based on the Ningbo Eye Hospital as the leader and the community health service center, the trial operation was carried out for 2 years, 2000 cases were collected, and manual work was carried out at the same time. Reading and Dr automatic screening: assign the same ophthalmologist to make manual judgment to judge the performance of Dr automatic screening system based on nonmydriatic fundus images. Count the screening results, that is, the image of the fundus of the sugar net, the image of the healthy fundus, the number of DR, and the number of healthy people. At the same time, it is compared with the manual judgment result to calculate the accuracy and processing efficiency. Assess the level of filming and diagnosis at the grassroots level: hold training classes for grassroots community doctors to improve the level of fundus photo shooting of grassroots doctors, and regularly send experts from Ningbo Eye Hospital to the grassroots to guide and conduct work; in addition, the skill assessment and scoring of primary doctors will be conducted every 2 months for 2 years. Regularly analyze and record the image quality parameters taken by the grassroots doctors in the community, including the characteristics of image color, focus, contrast, and illuminance, to judge and assess the level of fundus photography of the grassroots doctors in the community. Select 10 grassroots community doctors in the medical union, evaluate the diagnosis level of grassroots community doctors every six months during the project, and follow up and analyze it for a long time.

## 4. Experiment and Analysis

### 4.1. Data Collection and Preprocessing

This part integrates medical data mining theory with real-world experience from a Ningbo Eye Hospital to integrate and preprocess medical data. Integrating the patient's medical record information can not only facilitate the analysis of pathological information by doctors, but also provide data support for the research of intelligent diagnosis of diabetes. In order to ensure the effectiveness of the results of the system, the selected data are 2,265 electronic medical records in the past three years, and 2000 qualified medical records have been selected. Here are the following statistics: (1) gender ratio: 882 males and 1118 females and (2) proportion of age of patients: the oldest selected patient is 89 years old, the youngest is 19 years old, and the average age is 62.6 years. Most of them are between the ages of 60 and 70, with the 50 to 60 years old age bracket making up 23.5% of the total population. Among the 2000 patients, an expert classified 5 grades according to the severity of DR, namely nondiabetic retinopathy; mild proliferative diabetic retinopathy; moderate nonproliferative diabetic retinopathy; severe nonproliferative diabetic retinopathy; and proliferative diabetic retinopathy. Among them, 60% of the cases are used as the training set, and 40% are used as the test set.

### 4.2. BP Network Parameter Selection and Structure Design

A vast number of neurons in the network are connected to each other, and part of the calculation is done independently before the information processing is completed in collaboration. The BP neural network has excellent fault tolerance. The BP network's information and data are broken down into innumerable units and stored in various locations throughout the world. Because of this construction, even if a unit is damaged, it will have little effect on the overall operational outcomes. As the training progresses, the BP neural network's weights will be changed. As the weights rise, the neural connections get stronger, increasing the BP network's sensitivity to this trait. Electronic medical records often contain data that are dispersed and incomplete. From them, effective information is tough to wrest. In medical data analysis, BP neural network's collaborative processing and quick computation capabilities come in handy. The building of the neural network, training, and diagnosis phases are all included in a diagnosis model based on the BP neural network. Normalize the sample data, normalize the sample to the interval [−1, 1] to improve the network training speed, adopt *x*′=*x* − min*A*/max*A* − min*A*, and max*A* and min*A* are the maximum and minimum attributes, respectively.

In this paper, in order to enable the system to learn quickly and stably, the learning rate LR is selected as 0.01. If the learning rate is too small, it will not only reduce the learning rate, but also increase the instability of the network. In order to increase the diagnostic accuracy, the target error is selected as 0.01, and the Levenberg–Marquardt method is used as the training function. Hidden layer and output layer adopt *S*-type function and bipolar *S*-type function:

(6) $$\begin{array}{c} \text{log sig}\left(x\right)=\frac{1}{1+e^{-ax}},\\ \text{tan sig}\left(x\right)=\frac{2}{1+e^{-ax}}-1, \end{array}$$

where the value range is (0,1).

Using a three-layer BP network, it is possible to perform n-to-m-dimensional mappings quickly. Even if you increase the number of hidden layers, you will not see any change in the overall network's computational complexity. There is currently no quantitative standard for the selection of the number of hidden layer units, and it is usually used $h=\sqrt{n+m}+a,\;a\in \left(1,10\right)$ to determine the number of hidden layer units. In this study, *n* is 10 and *m* is 5. It is preliminarily determined that the range of the number of hidden layer units in this model is [4–14]. Therefore, this article takes 4, 6, 8, 10, 12 as the number of neurons in the hidden layer, uniformly covers the entire value range, and observes the training process, as shown from Figures 3–7.

According to Figures 3–7, there are stronger training effects and more network iterations when the number of hidden layer units is 10. As a result, for the sake of BP neural network modeling, this research opts for 10 hidden layer units. The BP neural network fits the data the best when it includes 10 hidden layer units, as illustrated in Figure 8, which shows a sample regression coefficient.

Among the 2000 patient data selected, the total number of data used as the training set is 1200, divided into 120 groups. There are 800 cases of data used as the test set, divided into 80 groups. The output results after BP neural network training and testing are shown in Table 1. The experimental results show that it is feasible to use BP neural network for DR diagnosis.

### 4.3. Comparative Analysis of the Accuracy of the Two Paths

Among the 80 sets of test data, 4 sets of data were misdiagnosed in the data diagnosed by a fundus specialist, with an average diagnosis accuracy rate of 95%. Comparing the time taken by the two paths, the time taken by artificial intelligence screening is 1/20 of the time taken by a fundus specialist.

The diagnostic accuracy rates of the manual screening and BP model after 80 tests are shown in Table 2. In order to further quantitatively compare the diagnostic accuracy rates of the two models, the average accuracy rate and the corresponding standard deviation of the test are calculated. It can be seen that the two paths have shown good results in the diagnosis of DR, but under the same conditions, the BP network model is higher than manual screening, and the efficiency is higher.

## 5. Conclusion

In recent years, the enthusiasm for the development of smart medicine at home and abroad has continued to increase. On the one hand, breakthroughs in key technologies such as image recognition, deep learning, and neural networks have brought about a new round of development in artificial intelligence technology. On the other hand, with the continuous improvement of people's living standards, the incidence of DR in China has also continued to rise, but in reality, there are problems such as uneven distribution of medical resources, insufficient number of doctors, and the level of community doctors that are far from top doctors. In order to allocate medical resources more effectively and reduce misdiagnosis due to lack of experience, this article combines artificial intelligence technology with DR diagnosis to help doctors diagnose DR. The main work and conclusions of this paper are as follows: (1) diabetes data collation. Based on medical data mining knowledge, this paper collected 2,265 electronic medical records from an eye hospital in Ningbo and selected 2,000 qualified medical records for data integration and preprocessing. The contents of electronic medical records mainly include age, gender, and examination records. (2) Establish DR diagnosis model based on neural network algorithm. This article first uses the classic algorithm of BP neural network to model. In the process of model building, the sample data are normalized. In order to enable the system to learn quickly and stably, the learning rate IR is selected as 0.01. In order to increase the diagnostic accuracy, the target error is selected as 0.01, the Levenberg–Marquardt method is selected as the training function, and the number of hidden layer units is selected as 10 through comparison experiments. Then, 80 sets of test data were diagnosed by ophthalmologists, and the correct rate of diagnosis was obtained. Finally, this paper compares and analyzes the accuracy of the two paths in 80 tests and concludes that the BP network model is superior to manual screening in terms of performance and accuracy.

## Figures and Tables

**Figure 1:** Two-layer forward neural network.  *f* is the transfer function, *x* is the input, *W* is the weight, and *y* is the output.

**Figure 2:** Controlled research technology roadmap.

**Figure 3:** Training effect when *N* = 4.

**Figure 4:** Training effect when *N* = 6.

**Figure 5:** Training effect when *N* = 8.

**Figure 6:** Training effect when *N* = 10.

**Figure 7:** Training effect when *N* = 12.

**Figure 8:** When *N* = 10, sample regression situation.

**Table 1:** BP neural network test results.

BP neural network	Diagnosed	Misdiagnosed	Accuracy (%)
Training result	116	4	96.67
Test result	77	3	96.25

**Table 2:** Comparison of accuracy and standard deviation between the two methods.

Method	Diagnosed	Misdiagnosed	Acc (%)	Standard deviation
BP neural network	77	3	96.25	1.25
Manual screening	76	4	95	2.68

## Data Availability

The data sets used and analyzed during the current study are available from the corresponding author upon reasonable request.
